# Contemporary management of fibrolamellar hepatocellular carcinoma: diagnosis, treatment, outcome, prognostic factors, and recent developments

**DOI:** 10.1186/s12957-016-0903-8

**Published:** 2016-05-23

**Authors:** Woubet Tefera Kassahun

**Affiliations:** Department of Surgery II, Faculty of Medicine, Clinic for Visceral, Transplantation, Thoracic and Vascular Surgery, OKL, University of Leipzig, Liebig Strasse 20, 04103 Leipzig, Germany

**Keywords:** Fibrolamellar hepatocellular carcinoma, Conventional hepatocellular carcinoma, Liver resection, Liver transplantation, Clinical outcome

## Abstract

Fibrolamellar hepatocellular carcinoma (FL-HCC) is a malignant liver tumor which is thought to be a variant of conventional hepatocellular carcinoma (HCC). It accounts for a small proportion of HCC cases and occurs in a distinctly different group of patients which are young and usually not in the setting of chronic liver disease. The diagnosis of FL-HCC requires the integration of clinical information, imaging studies, and histology. In terms of the treatment options, the only potentially curative treatment option for patients who have resectable disease is surgery either liver resection (LR) or liver transplantation (LT). When performed in a context of aggressive therapy, long-term outcomes after surgery, particularly liver resection for FL-HCC, were favorable. The clinical outcome of patients with unresectable disease is suboptimal with median survival of less than 12 months. The aim of this review is to update the available evidence on diagnosis, treatment options, outcome predictors, and recent developments of patients with this rare disease and to provide a summarized overview of the available literature.

## Background

Fibrolamellar hepatocellular carcinoma (FL-HCC) is thought to be a rare variant of conventional hepatocellular carcinoma (HCC), accounting for 0.85 to 16 % of all hepatocellular carcinomas [1–7]. It occurs in a distinctly different group of patients which are young and usually not in the setting of chronic liver disease (Table 1). The majority of such cases offer vague and nonspecific clinical symptoms, including weight loss, fatigue, abdominal pain, and a mass lesion. Alternatively, patients can be asymptomatic and had their disease discovered incidentally during diagnostic workup of an unrelated medical condition. Thus, the biological behavior of FL-HCC can range from an indolent, clinically insignificant disease to an aggressive pattern of locally invasive disease or distant metastasis [1, 4, 6, 8–10]. The main goal in the assessment of patients with FL-HCC is to distinguish FL-HCC from other malignancies of the liver particularly HCC and liver metastases and other benign liver lesions such as focal nodular hyperplasia (FNH) and hepatocellular adenoma (HCA). This requires the integration of clinical information with conventional diagnostic techniques such as ultrasound (US), computed tomography (CT) scans, magnetic resonance imaging (MRI), and histology. The only potentially curative treatment option for patients who have resectable disease is surgery either liver resection (LR) or liver transplantation (LT). Because it is increasingly safe and offers a truly curative therapy, liver resection remains the standard of care for patients with locoregional disease in a non-cirrhotic liver. When performed in a context of aggressive therapy, long-term outcomes after surgery, particularly liver resection for FL-HCC, were favorable. Unfortunately, disease recurrence is high, at 33–100 % [11]. Even after curative-intent surgery, disease recurrence is frequent, often in the first 4 years postsurgical [12]. However, it can also occur after 5 years or even longer [6, 11]. Thus, after treatment for FL-HCC, prolonged follow-up is necessary because recurrence and death can occur years after diagnosis. For patients with resectable FL-HCC, 5-year survival rates as high as 80 % and 5-year disease-free survival rates of 18 to 50 % have been reported (Table 2). The clinical outcome of patients with unresectable disease is suboptimal with median survival of only 12 months and no patient surviving beyond 5 years [6, 10]. Furthermore, the role of neoadjuvant and adjuvant therapies, including systemic chemotherapy and radiotherapy, remains poorly defined and has been reported to have only a modest or no therapeutic effect [2, 10, 13]. Reports on the characteristics of patients with FL-HCC as well as predictors of recurrence and survival are scarce, probably due to the rarity of this tumor, and are limited to case series, small cohorts, and few systematic reviews. The aim of this review is to update the available evidence on diagnosis, treatment options, and outcome of patients with this rare disease and to provide a summarized overview of the available literature.

**Table 1:** Clinicopathologic characteristic of fibrolamellar hepatocellular carcinoma in comparison to conventional hepatocellular carcinoma

Characteristic	FL-HCC	HCC	Comments
Age at presentation	Young	Older	
Sex predilection	No	4–8 times more often in men	
Distinct geographic distribution	No	Yes	HCC is more often seen in Africa and Asia
Distribution of lesions	Mostly solitary	Mostly multiple	
Growth pattern	Indolent	Aggressive	
Stage at diagnosis	Mostly advanced	Mostly advanced	Despite the advanced stage at diagnosis, prognosis is in favor of FL-HCC patients
Chronic viral infection	Absent	Present	
Liver cirrhosis	Absent	Present	Occasionally, underlying liver disease may be present in patients with FL-HCC. If present, incidental and not causative for FL-HCC
α-fetoprotein	Within normal range	Mostly elevated	
Liver resection	Treatment of choice	Not standard	Limited indication in HCC due to cirrhosis
Liver transplantation	Not standard	Curative treatment	If requirements for LT are fulfilled
Prognosis	Favorable	Mostly dismal	No difference in non-cirrhotic patients
Macro-finding	Well-circumscribed, often lobulated mass, a central gray and white scare	Single or massive, multifocal or nodular, and diffuse. Due to lack of stroma in the tumor, often necrosis and hemorrhage	
Histology	Eosinophilic polygonal-shaped cells separated by lamellar fibrosis. A fairly uniform cell pattern. Overall, greater differentiation than HCC	Thickened plates of hepatocytes with eosinophilic or clear cytoplasm. Cells are often arranged in trabecular, pseudoglandular, or solid pattern	Histologic appearances are the most objective and widely accepted differences between FL-HCC and HCC

*FL-HCC* fibrolamillar hepatocellular carcinoma, *HCC* conventional hepatocellular carcinoma

**Table 2:** Summary of clinicopathologic and outcome data of patients with fibrolamellar carcinoma collected from the literature

Author	TP	YP	Total number of patients	♂:♀	Age	CD %	AFP↑	LR %	LT %	5y-OS %, LR	5y-OS %, LT	DR %	5y-DSF %	5y-OS %
Craig et al. [8]	1918–1973	1980	23	1:1	26	None	0/6	48	None	nr	na	nr	nr	nr (32)
Nagorney et al. [9]	1950–1982	1985	16	1.3:1	26	None	1/6	75	None	nr	na	75	42	50
Berman et al. [17]	1981–1987	1988	19	2.2:1	25	None	4/15	63	26	nr	nr	59	nr	nr (37)
Wood et al. [51]	1960–1983	1988	15	1:2.8	26	None	3/9	60	None	45	na	nr	nr	45 (32)
Iwatsuki et al. [68]	1980–1989	1991	22	nr	nr	nr	nr	55	45	65	38	nr	nr	nr
Ringe et al. [1]	1974–1988	1992	20	1.2:1	23	None	0/18	70	30	40 (45)	nr (29)	60	29	37 (45)
Pinna et al. [2]	1968–1995	1997	41	1.3:1	30	7	2/19	68	32	75	36	66	33	66 (127)
Epstein et al. [30]	1985–1990	1999	17	1:1	24	None	0/16	None	None	na	na	nr	na	nr (14)
El-Gazzaz et al. [3]	1985–1998	2000	20	1:1.9	27	None	0/20	55	45	65	50	45	50	50 (62)
Ichikawa et al. [14]	1989–1997	2000	40	1:1.2	29	None	3/40	62	10	nr	nr	71	nr	nr
El-Serag and Davila [4]	1986–2000	2004	68	1:1	33	nr	nr	nr	nr	nr	nr	nr	nr	37
Kakar et al. [10]	1987–2000	2005	20	1:1	27	None	3/13	nr	nr	nr	nr	nr	nr	45
Moreno-Luna et al. [5]	1990–2003	2005	15	nr	nr	nr	nr	80	None	nr	na	nr	nr	26
Stipa et al. [6]	1986–2003	2006	41	1:1.4	27	None	3/41	68	None	76	na	61	18	76 (112)
Malouf et al. [23]	1987–2007	2012	40	0.3:1	22	3	7/40	100	None	58	na	58	37	58
Mavros et al. [11]	1963–2008	2012	575	1:1.1	21	3	27/266	55	23	70 (222)	34 (32)	33–100	nr	44 (39)
Ang et al. [58]	1986–2011	2013	95	0.7:1	22	nr	3/31	73	4	nr	nr	77	nr	nr
Kaseb et al. [7]	1992–2008	2013	94	1:1	23	6	13/94	59	2	nr	nr	84	nr	46 (57)
Eggert et al. [69]	2000–2010	2013	191	1.7:1	nr	nr	nr	41	46	58	57	nr	nr	34
Groeschl et al. [12]	1993–2010	2014	35	1.7:1	39	14	1/35	100	None	62	na	50	45	62 (174)
Darcy et al. [15]	1981–2011	2015	25	1:1.3	17	None	2/25	84	None	52	na	63	nr	43

*TP* time period, *YP* year of publication, *♂:♀* male to female ratio, *CD* number of patients with chronic liver disease particularly liver cirrhosis in percent of the total number of patients, *AFP↑* number of patients with pathologic elevation of alpha-fetoprotein in relation to tested patients, *LR* liver resection, *LT* liver transplantation, *5y-OS* 5-year overall survival (numbers in bracket indicate the average survival in months for any treatment), *DR* disease recurrence, *DSF* disease free survival, *nr* not reported, *na* not applicable

## Review

### Diagnosis

#### Clinical finding

Diagnosis of FL-HCC requires consideration of the clinical conditions, imaging studies, and histologic evaluation. Patients with FL-HCC are typically young, without underlying liver disease, and asymptomatic. Therefore, this tumor forms a difficult problem in diagnosis. When patients with FL-HCC are symptomatic, they typically present with nonspecific abdominal pain or discomfort, weight loss, a palpable liver mass, ascites, and lower edema [3, 5, 14]. There may also be a constellation of symptoms, including anorexia, fever, and jaundice, and this subject has been recently reviewed by Darcy et al. [15]. These authors reported that the most common presenting symptom is abdominal pain (72 %) followed by abdominal distention (44 %), anorexia (32 %), fever, and jaundice (20 %). Craig et al. 1980 [8] reported that abdominal pain as the main presenting symptom is highly variable in duration ranging from 1 to more than 6 months preceding the diagnosis of FL-HCC. In general, symptoms are usually present 3 to 12 months before diagnosis [16].

The routine biochemical and hematological values of FL-HCC patients are mostly normal or mildly elevated in a nonspecific fashion [1, 17].

### The role of tumor markers

Alpha-fetoprotein (AFP) is the most well-studied serum marker widely used in diagnostic and screening of HCC. Unlike HCC, FL-HCC rarely produces AFP. Consequently, patients with FL-HCC rarely have elevated serum levels of AFP, and AFP has been demonstrated only in the minority of patients with FL-HCC in the tumor immunohistochemically [17]. Elevated levels of serum vitamin B_12_- and serum unsaturated vitamin B_12_-binding capacities have been described as associated with FL-HCC by some authors [18, 19]. However, additional evidence and experience are needed to determine the strength of this association. Elevated serum neurotensin was found to have a role as a biomarker in some cases, but did not prove to be sensitive or specific enough for diagnosis [15, 20].

### Imaging diagnostic

Imaging of the liver which is an integral part of every diagnosis is largely performed by cross-sectional imaging modalities including US, CT, and MRI.

Nuclear medicine studies such as FDG PET can be utilized once a liver lesion is detected and/or there is a clinical suspicion for extrahepatic manifestation and may be helpful in narrowing the differential diagnosis. However, the role of nuclear medicine in the imaging diagnostic of FL-HCC has not been fully evaluated [21].

Thus, when a liver mass is detected, characterization can be performed by several different imaging techniques. Multiphasic examinations are required with acquisition of images before and dynamically after the administration of contrast media to characterize the mass and to determine the extent of disease. In general, the technique employed is usually determined by institutional preference and experience as well as other clinical factors such as patient history and comorbid conditions such as kidney failure. US is the initial diagnostic modality for evaluating the liver. It can detect an intrahepatic mass and intrahepatic or extrahepatic ductal dilation. However, US is nonspecific and less accurate than CT or MRI to differentiate FL-HCC from other mass-forming lesions of the liver. Although CT is adequate for initial pretreatment imaging of FL-HCC, particularly for evaluation of metastatic lesions, MRI may be helpful for initial workup when FL-HCC is first discovered as an initial liver mass [22]. In general, FL-HCC tends to present as a large, heterogeneous enhancing mass that may contain a central scar and/or calcifications on imaging. Details about imaging findings have been reviewed extensively in previous publications [14, 16, 21–29] and summarized in Table 3. Portal vein thrombosis and biliary obstruction are extremely rare occurring in only 5–10 % of cases [14, 16, 23, 26, 28]. Nodal metastatic lesions are most commonly seen at the hepatic hilum and hepatodudenal ligament occurring in up to 50 to 60 % of cases [6, 14, 21]. Distant metastatic disease from FL-HCC, mostly to the lungs, peritoneum, and adrenal gland has been reported on imaging in up to 20–30 % of cases [4, 21, 30].

**Table 3:** Summary of diagnostic imaging findings [14, 16, 22–29, 31]

Diagnostic imaging	Finding FL-HCC	Finding HCC in cirrhosis	Comments
US	- Well-defined mass of variable echogenicity - Partially successful in demonstrating central scares as a central area of hyperechogenicity - Demonstrates calcification within the fibrous scar	- Lesions may appear hyperechoic, hypoechoic, or as target lesions, none of which is specific	- In general, nonspecific sonographic features - Less useful for demonstrating necrosis - Less accurate than CT and MRI in demonstrating regional lymphadenopathy - The optimal tool for screening HCC in cirrhosis
CT	- Large tumor with well-defined margins - Lobulated or smooth surface - Calcification and a central scare - Areas of hypervascularity - Abnormal lymphadenopathy - Portal vein thrombosis and biliary obstruction are extremely rare - Generally tumors show a heterogeneous hypervascular enhancement	- Necrosis, hemorrhage, focal tumor fat, and invasion of vascular structures are common - Hypoattenuating to surrounding liver - Central scare, fibrosis, and calcification are rare - Arterial hypervascularity (elevated arterial flow), venous phase washout (reduced or absent portal venous flow) - Presence of fat	- In some cases of FL-HCC margins can be ill defined. - CT demonstrates calcification in FL-HCC better than MRI. - In CT a central scare is not pathognomonic of FL-HCC
MRI	- Large tumor, hypointense on T1-weighted images and hyperintense on T2-weighted images - No calcification but a central scare - No fat component - Generally tumors show a heterogeneous hypervascular enhancement; hyperattenuating on the arterial phase, hypo-, iso-, or even hyperattenuating in venous phases	- Well-circumscribed borders - Low signal intensity on T1-weighted images and high signal intensity on T2-weighted images - Intratumoral fat - Tumor encapsulation - Portal or hepatic vein invasion - Arterial-portal venous shanting - Generally, variable in appearance depending on steatosis or hemorrhage	- MRI is considered to be competitive rather than complimentary to CT in most cases. - MRI demonstrates the central scare in FL-HCC better than CT - MRI is may be more sensitive in detecting small lesions

*FL-HCC* fibrolamellar hepatocellular carcinoma, *HCC*, usual hepatocellular carcinoma, *US* ultrasound, *CT* computed tomography, *MRI* magnetic resonance imaging

### The role of biopsy

Histologic appearances are the most objective and widely accepted differences between FL-HCC and HCC [31, 32]. Therefore, histologic confirmation is needed to be able to diagnose FL-HCC with certainty. This is particularly important if there is diagnostic uncertainty about the imaging diagnosis. It enhances the ability to select patients properly for aggressive surgical intervention by excluding the subset of patients who do not appear to benefit from surgical therapy, such as those with extensive metastatic disease or with underlying medical conditions that preclude surgery. Fine needle aspiration has low yields and may aspirate malignant hepatocytes without the characteristic fibrotic lamellae resulting in a diagnosis of HCC and not FL-HCC [33]. Thus, the preferred technique of biopsy is either percutaneous core biopsy or open biopsy via laparoscopy.

### Differential diagnosis

The differential diagnosis of FL-HCC includes a wide spectrum of nonneoplastic and neoplastic lesions of the liver such as FNH, HCA, and HCC [34]. Differentiation of other liver lesions from FL-HCC permits optimal patient treatment. Some of these entities may show characteristic imaging findings including morphology that permit their diagnosis (Table 4). However, radiologic findings are generally inconclusive for a differential diagnosis because the appearance of the lesions on the various imaging studies of FL-HCC patients may closely simulate that of FNH, HCA, HCC, or metastasis [29]. Correlation with clinical and demographic data may help narrow the differential diagnosis in patients with FL-HCC. Overall, however, biopsy may be required to achieve definitive histopathologic characterization in most cases.

**Table 4:** Clinicopathologic and imaging characteristic of fibrolamillar hepatocellular carcinoma in comparison to focal nodular hyperplasia and hepatocellular adenoma [21, 35–45, 70–72]

Lesion Characteristics	FL-HCC	FNH	HCA
Entity	Malignant	Benign, mainly proliferating normal hepatocytes	Benign with the potential to malignant transformation
Location	Anywhere in the liver	Frequently in the periphery	Anywhere in the liver
Size and number	Single, large, and lobulated	Single or multiple, small in size	Single or multiple, small in size
Sex predilection	No	Otherwise healthy young women	Otherwise healthy young women
Causal relationship to oral contraception (OC)	Not known	Not known	Yes
Main findings on imaging	CT: large tumor, heterogeneous hypervascular enhancement MRI: Large tumor, hypointense on T1-weighted and hyperintense on T2-weighted images, T2 hypointense central scare, no fat component, hyperattenuating on the arterial phase, hypo-, iso-, or even hyperattenuating in venous phases	CT: arterial enhancement, presence of central scare MRI: arterial enhancement, central scare predominantly T2 hyperintense, homogeneous signal intensity, accumulation of liver-specific contrast agent within the central area on delayed T1 images	CT: arterial enhancement, precontrast hyperdense areas showing hemorrhage, low-density areas showing necrosis or fat MRI: arterial enhancement, hyperintense areas on T1, T2 images showing hemorrhage, hypointense areas on T1 that correlate to hyperintense areas on T2 images showing necrosis, no accumulation of liver-specific contrast agent within the lesion
Treatment	Surgical	Normally requires no treatment	Discontinuation of OC, surgical

*FL-HCC* fibrolamellar hepatocellular carcinoma, *FNH* focal nodular hyperplasia, *HCA* hepatocellular adenoma, *CT* computed tomography, *MRI* magnetic resonance imaging

### Focal nodular hyperplasia

Focal nodular hyperplasia is a hyperplastic nodule that contains scar-like tissue [35]. It is believed to originate from hepatocyte proliferation around a congenital arteriovenous malformation and is the second most common benign hepatic lesion after hemangioma, mostly seen in women and incidentally detected [36, 37]. Its growth is may be promoted by oral contraception (OC) but has no evidenced causal relationship to OC. Because of macroscopic similarities, common age, and gender to FL-HCC, FNH is often confused for FL-HCC [33]. Distinction between these two diagnoses is important because the clinical approach regarding both is different. While surgery is the treatment option for patients with FL-HCC, patients with FNH does not require treatment.

### Hepatocellular adenoma

Hepatocellular adenoma is a rare benign neoplasm of the liver that occurs typically in young women of child-bearing age who have a long history of estrogen-based oral contraceptive use [38, 39]. Owing to hormone-induced growth, these lesions may rupture and bleed spontaneously leading to massive hemorrhage [40]. Besides the risk of rupture and bleeding, about 4.2 % of HCAs have the potential to undergo malignant transformation into HCC [41]. Thus, the preferred treatment option is liver resection particularly if lesions are >5 cm in diameter [42]. The diagnosis of HCA is usually made based on the clinical and imaging findings and the findings of core biopsies obtained for diagnostic workup of a liver mass [33, 43–45]. However, HCA may sometimes show overlapping diagnostic features with FL-HCC posing a diagnostic challenge.

### Hepatocellular carcinoma

There are major differences in the clinicopathologic characteristics between conventional HCC and its variant FL-HCC (Table 1). HCC accounts for significant global morbidity and mortality, especially in endemic areas of chronic viral infection [46]. Contrary to FL-HCC, HCC has well-defined major risk factors such as chronic viral infection with hepatitis B and C and aflatoxin B1 intake with contaminated food that lead to liver cirrhosis [47–49]. The majority of cases of HCC develop in liver cirrhosis, making liver cirrhosis the strongest predisposing factor [50]. Furthermore, HCC predominantly occurs in older patients with significant sex predilection (more often in men over the age of 60), whereas FL-HCC typically affects adolescents and young adults with a nearly even sex distribution [19, 21].

### Surgical treatment

Data in the literature shows that patients with FL-HCC are good candidates for aggressive surgical treatment; these patients can expect a reasonable likelihood of durable survival [12]. Liver resection and liver transplantation are aggressive approaches to the treatment of patients for FL-HCC and are the only known potentially curative treatment options for this tumor.

### Liver resection

Liver resection is the treatment of choice for FL-HCC unless it arises in the setting of liver cirrhosis which is extremely rare. In the absence of liver cirrhosis, patients with FL-HCC have a high resectability rate (Table 2). As the majority of FL-HCC patients are young and otherwise healthy, major liver resection can be done with low rates of life-threatening complications [46]. Multiple studies demonstrated OS of 26–76 % at 5 years with a median survival of 32–174 months for resected patients [1–3, 6, 7, 11, 12, 51]. Five-year recurrence-free survival was as low as 18 %; however, even patients in advanced stage including those with disease recurrence seem to benefit from aggressive surgery. For example, despite the fact that 90 % of their patients presented with stage IV disease, Pinna et al. [2] reported an overall actuarial survival of 66 % at 5 years and 47 % at 10 years. According to these authors, this survival advantage was attributed to indolent growth, favorable biological behavior, and suitability to extensive liver resection including adjacent structures initially as well as to treat recurrence.

Disease recurrence after complete surgical resection is high in this patient population ranging 33–100 % [1–3, 7, 9, 11–15]. The median time to recurrence is relatively short at between 10 and 33 months [1, 3, 6, 13, 14]. However, recurrence of disease more than 5 years after surgery is a rare event [2, 12]. The high recurrence rate after surgery may seem somewhat surprising, especially given that patients were treated aggressively and at highly specialized hepatobiliary centers. However, quite often patients with FL-HCC are referred to these centers at an advanced stage, with large primary tumors and evidence of lymph node metastases, both factors which has been identified as negative prognostic indicators [2, 3, 6, 12, 13, 15]. Furthermore, for those patients with recurrence after liver transplantation, in addition to advanced tumor stage, the issue of immunosuppression should also be considered because it may significantly increase the recurrence rate [52].

Repeat surgery has been considered by many to be the most effective treatment for recurrence [6–8, 12]. Re-resection aimed at recurrent or metastatic disease, when possible, may provide patients with good long-term results. For example, in a study of Stipa et al. [6], 28 patients with FL-HCC underwent LR with an overall recurrence rate of 61 %. The mean time to recurrence was 37 months. Recurrence was exclusively intrahepatic in approximately half of the 17 patients with disease recurrence. Despite this high recurrence rate, all patients were amenable to treatment with re-resection that resulted in median survival of 26 months. In the study of Kaseb et al. [7], metastasectomy was done in 18 cases and was found to be significantly associated with longer OS. The median OS was 145 months for those who underwent surgery versus 35 months for those who did not. In the study of Maniaci et al. [13] that included 10 patients, disease recurrence occurred in all patients following initial surgery with a median time to recurrence of 2.2 years. In seven patients, disease recurrence was managed surgically that resulted in a median survival of 4.7 years and an OS of 48 % at 5 years. Therefore, as such, tumor recurrence should not preclude resection when complete removal can be achieved because it carries a relatively good prognosis. Patient selection and an emphasis on surgical technique to achieve complete removal are pivotal to optimizing the best chance for the best possible outcome.

### Liver transplantation

LT is an effective treatment for HCC, and its indications are expanding [53]. On the contrary, only FL-HCC which is not amenable to resection but confined to the liver is considered a suitable indication for LT by the majority of investigators [2, 3, 11]. Thus, the use of LT for advanced disease is unique to FL-HCC. However, owing to its rarity and the infrequent need for LT, available data is limited. Theoretically, LT has the potential to readily achieve a clean margin, accomplish a radical removal of the tumor, and treat underlying liver disease when present. In 1997, Pinna et al. [2] examined the results of 13 patients who underwent LT for FL-HCC. The overall 3- and 5-year survival rates were 45 and 36 %, respectively. However, disease recurrence was confirmed in 9 (69 %) out of 13 Patients. These authors analyzed the specific factors that might serve as predictors of disease recurrence after LT. Patients with regional lymph node involvement (N1), those with the presence of metastasis (M1), and those with stage IVB disease were more likely to develop recurrent disease. Interestingly, the use of chemotherapy in an adjuvant setting was also associated with earlier intrahepatic recurrence.

In a series which included nine patients with FL-HCC treated by LT, El-Gazzaz et al. [3] reported 1-, 3-, and 5-year survival rates of 90, 75, and 50 %, respectively. Disease recurrence occurred in five (56 %) out of nine transplanted patients. Two of the nine transplanted patients received chemotherapy in neoadjuvant and adjuvant setting, and chemotherapy had no detectable effect on survival or recurrence-free survival.

In a systematic review published in 2012, Mavros et al. [11] reported the results of 14 studies that included 109 patients after LT for FL-HCC. Six studies reported specific survival data on 79 patients. Survival after 1, 3, and 5 years ranged from 63 to 100 %, 43 to 75 %, and 29 to 55 %.

In a meta-analysis of 17 studies involving 368 patients with FL-HCC and 9877 patients with conventional HCC, Njei et al. [54] found significantly higher 5-year survival rates in those patients with FL-HCC treated by LR than did those with conventional HCC. But, they found no difference in survival in patients undergoing liver transplantation.

Overall, patients who underwent LR for FL-HCC did better than patients who underwent LT. However, with the number of published trials increasing, the aggregate data indicated acceptable outcomes for patients who underwent LT as well. Thus, given the advanced stage of disease in transplanted patients, LT for FL-HCC does not appear to be an inferior treatment option in comparison with LR and may have more indications than the current standard of care. However, given the rarity of the disease and the retrospective nature of data collection from different institutions with a very small sample size, most published series lack sufficient power for statistical analysis and the results are inconclusive. Thus, the perception of good survival outcomes after LT despite the advanced stage of disease is probably inaccurate and should therefore be interpreted with caution.

### Chemotherapy

The role of neoadjuvant or adjuvant chemotherapy is controversial. In some cases, chemotherapy had no effect on survival or recurrence in patients who received chemotherapy after surgery [2, 3]. Contrary to this, in other studies, patients who had chemotherapy in neoadjuvant and adjuvant settings fared better than those with surgery only with patients who had front-line surgery followed by chemotherapy having the longest OS [7, 55]. In one report [56], the use of platinum-based chemotherapy in pediatric patients with FL-HCC resulted a partial response in 31 % of patients on imaging but a 3-year survival of only 22 %. Thus, although some different types of systemic chemotherapy for FL-HCC have been tried, the advances in tumor downstaging with this therapeutic option have not proven effective. The most difficult aspect of understanding the utility of chemotherapy for FL-HCC is that no prospective trials have investigated different types of chemotherapy options. Instead, most knowledge about the effectiveness of chemotherapy is based on anecdotal evidence and single-patient experience.

### Outcome and prognostic factors

Although FL-HCC patients often present with an advanced disease, approximately 50–84 % of affected patients are amenable to surgical treatment and have an OS as high as 76 % at 5 years (Table 2). Thus, patients with FL-HCC appear to have a better prognosis than those with HCC which have a far worse prognosis with a 5-year survival of only 6.8 % [4]. However, considering similar stage disease, patients with FL-HCC do not have a favorable prognosis and do not respond any differently to treatment than patients with HCC in non-cirrhotic livers [9, 10, 51, 54, 57]. This suggests that the apparent better outcome seen in FL-HCC may be related to the absence of liver cirrhosis. Thus, as indicated by some of the reviewed studies, along with the indolent nature of the disease and younger age, the most likely reason for this favorable outcome is the absence of liver cirrhosis that allows aggressive surgical treatment [4, 6, 8, 10, 17]. Individual tumor stage, number and size of tumors, vascular invasion, regional lymph node metastasis, the presence of extrahepatic disease, non-White race, and female gender have been thought to be negative predictors of outcome after surgery [1, 2, 6, 10, 12, 15, 58]. Of these, the initial stage of the tumor at the time of treatment seems to be the most significant determinant of prognosis. Patients with stage I–III disease tended to fare better than patients with stage IV disease [1, 2, 6, 23], and in some cases, this difference attains statistical significance [2, 12, 23]. Overall, however, additional studies with large number of patients are needed, since the existing data does not result in a differentiation firm enough to base treatment decisions on.

### Recent developments

Currently, researchers are attempting to provide some insights into the molecular characteristics of FL-HCC. Using genomic analysis, some patterns of genomic aberrations which are different from other liver malignancies have been shown and possible pathways and candidate genes as therapeutic targets have been identified. However, these discoveries of molecular pathways and genetic mutations that characterize FL-HCC have not yet enhanced the ability to design specific anticancer therapies.

DNAJB1-PRKACA: this recently described predominant fusion protein has been proved to retain the kinase activity of PRKACA, the catalytic subunit of protein kinase A (PKA) [59–61]. DNAJB1-PRKACA may represent a potential therapeutic target as high levels of DNAJB1-PRKACA protein expression (amplified in more than 70 % of FL-HCC) have been found in FL-HCC compared to a normal liver or HCC [59]. Because of the many oncogenic signaling pathways regulated by PKA [62, 63], kinase inhibitors which bind near the active site of the PKA catalytic subunit can target several oncogenic proteins in parallel [64]. Currently, however, no known drug trials are using such inhibitors specifically against FL-HCC.

mTOR: the mammalian target of rapamycin (mTOR) is an intracellular protein kinase (PK) expressed in mammalian cells and is critical in the development of many malignant tumors [65]. The mTOR pathway is responsible for regulating cell growth and survival. It mediates signaling transduction downstream of receptor tyrosine kinases. If this pathway becomes dysfunctional, mTOR becomes upregulated, leading to increased cell proliferation, angiogenesis, and evasion of apoptosis [66]. Consequently, inhibitors of this pathway have been assessed and evaluated for their safety and efficacy in cancer patients. For example, the mTOR inhibitor everolimus in combination with octereotide has been shown to be effective for low- and intermediate-grade neuroendocrine tumors. Most patients experienced either a partial response or stable disease, with a minority experiencing tumor progression [67].

Anticancer agents that induce durable remissions are needed particularly for those FL-HCC patients whose tumors are not amenable to aggressive surgery. Currently, it has been shown that mTOR signaling significantly activated in FL-HCC compared to other liver malignancies [61]. This suggests that mTOR inhibitors may have anticancer activity in FL-HCC as well. Recently, however, there have been no published trials using mTOR inhibitors that target its dysregulated pathways for patients diagnosed with FL-HCC. Thus, given the present results in drug research regarding the treatment of FL-HCC, it is highly unlikely that a marked prolongation of life in patients with advanced FL-HCC is on the immediate horizon.

## Conclusions

A familiarity with the diagnosis, treatment, and overall management of FL-HCC is necessary for all those dealing with these patients. The optimal approach to management involves accurate diagnosis and staging, followed by assessment of candidacy for liver resection or transplantation. The diagnosis of FL-HCC is often difficult, and it requires careful assessment of the clinical findings and multiple, complimentary, imaging modalities and biopsy. Liver resection is the preferred treatment option; however, in selected patients, liver transplantation can also be considered as an option. With few presented conflicting results of retrospective studies, the role of other therapeutic options such as chemotherapy is controversial. For now, it seems that these options are uniformly ineffective in prolonging survival. The resistance of FL-HCC to these treatment options likely contributes to poor outcomes in patients presenting with extensive metastatic disease. Surgery for recurrent disease, even when present with regional metastases, can achieve a meaningful survival benefit. Thus, surveillance must be maintained, even beyond 5 years. The more indolent course of this tumor and its good response to aggressive surgical therapy suggest that future research and treatment strategy should be designed in a manner that addresses more appropriately the treatment of patients who have tumors that may be less sensitive and not amenable to surgical therapy. Because of its very low incidence, research on targeted therapy is difficult and has not yet been successful. Therefore, national and international collaborations are required to achieve this objective.

## Ethics approval

Not applicable.

### Availability of data and materials

This manuscript is a literature review, and all used literature is referenced appropriately in the “References” section.

## Abbreviations

AFP: alpha-fetoprotein
FL-HCC: fibrolamellar hepatocellular carcinoma
FNH: focal nodular hyperplasia
HCA: hepatocellular adenoma
HCC: conventional hepatocellular carcinoma
LR: liver resection
LT: liver transplantation
